The article "Raf Kinase Inhibitor Protein (RKIP) Blocks Signal Transducer and Activator of Transcription 3 (STAT3) Activation in Breast and Prostate Cancer" was retracted in 2021. Reasons: manipulated images; duplicated images; original data or images not available; unreliable data.

# Raf Kinase Inhibitor Protein (RKIP) Blocks Signal Transducer and Activator of Transcription 3 (STAT3) Activation in Breast and Prostate Cancer

**DOI:** 10.1371/journal.pone.0092478

**Published:** 2014-03-21

**Authors:** Saad Yousuf, MeiLi Duan, Erika L. Moen, Sam Cross-Knorr, Kate Brilliant, Benjamin Bonavida, Theresa LaValle, Kam C. Yeung, Fahd Al-Mulla, Eugene Chin, Devasis Chatterjee

**Affiliations:** 1 Department of Medicine, Rhode Island Hospital and The Alpert Medical School of Brown University, Providence, Rhode Island, United States of America; 2 Department of Critical Care Medicine, Beijing Friendship Hospital, Capital Medical University, Beijing, China; 3 Department of Microbiology, Immunology and Molecular Genetics, University of California Los Angeles, Los Angeles, California, United States of America; 4 Kolltan Pharmaceuticals, Inc., New Haven, Connecticut, United States of America; 5 Department of Biochemistry and Cancer Biology, University of Toledo, College of Medicine, Toledo, Ohio, United States of America; 6 Department of Pathology, Faculty of Medicine, Kuwait University, Safat, Kuwait; 7 Department of Surgical Research, Rhode Island Hospital and The Alpert Medical School of Brown University, Providence, Rhode Island, United States of America; Thomas Jefferson University, United States of America

## Abstract

Raf kinase inhibitor protein (RKIP) is a member of the phosphatidylethanolamine-binding-protein (PEBP) family that modulates the action of many kinases involved in cellular growth, apoptosis, epithelial to mesenchymal transition, motility, invasion and metastasis. Previously, we described an inverse association between RKIP and signal transducers and activators of transcription 3 (STAT3) expression in gastric adenocarcinoma patients. In this study, we elucidated the mechanism by which RKIP regulates STAT3 activity in breast and prostate cancer cell lines. RKIP over expression inhibited c-Src auto-phosphorylation and activation, as well as IL-6-, JAK1 and 2-, and activated Raf-mediated STAT3 tyrosine and serine phosphorylation and subsequent activation. In MDA-231 breast cancer cells that stably over express RKIP, IL-6 treatment blocked STAT3 phosphorylation and transcriptional activation. Conversely, in RKIP knockdown MDA-231 cells: STAT3 phosphorylation and activation increased in comparison to parental MDA-231 cells. RKIP over expression resulted in constitutive physical interaction with STAT3 and blocked c-Src and STAT3 association. The treatment of DU145 prostate, but not PC3 prostate or MDA-231 breast, cancer cell lines with ENMD-1198 or MKC-1 dramatically increased expression of RKIP. Overexpression of RKIP sensitized PC3 and MDA-231 cells to MTI-induced apoptosis. Moreover, MTI treatment resulted in a decrease in Src-mediated STAT3 tyrosine phosphorylation and activation, an effect that was significantly enhanced by RKIP over expression. In stable RKIP over expressing MDA-231 cells, tumor xenograft growth induced by activated STAT3 is inhibited. RKIP synergizes with MTIs to induce apoptosis and inhibit STAT3 activation of breast and prostate cancer cells. RKIP plays a critical role in opposing the effects of pro-oncogenic STAT3 activation.

The article "Raf Kinase Inhibitor Protein (RKIP) Blocks Signal Transducer and Activator of Transcription 3 (STAT3) Activation in Breast and Prostate Cancer" was retracted in 2021. Reasons: manipulated images; duplicated images; original data or images not available; unreliable data.

## Introduction

Members of the signal transducer and activator of transcription (STAT) family are transcription factors located in the cytoplasm that, upon activation and nuclear translocation, regulate the expression of genes involved in cell growth, apoptosis, survival, and differentiation [1], [2]. Upon activation, STAT3 undergoes multiple posttranslational modifications, including phosphorylation and acetylation of STAT-family-conserved tyrosine, serine, and lysine residues in the carboxy-terminal region [3]–[6]. These specific modification events can be induced by treatment of cells with cytokines, growth factors, and hormones. Both Janus kinase (JAK) family and Src family tyrosine kinases can be recruited by cytokines or growth factor receptors to catalyze STAT3 tyrosine phosphorylation [7]–[10].

Cytokine/growth factor-activated STAT3 transcribes numerous genes that inhibit apoptosis and promote cell survival and neoplastic progression, including *bcl-XL*, *bcl-2*, and *mcl-1* [11], [12]; it also stimulates metastasis and invasion [13], [14]. Moreover, STAT3 is required for microtubule stabilization and stimulation of cell migration via inhibition of the microtubule-destabilizing Stathmin [15]. Aberrant JAK or Src protein kinase activity and constitutive STAT3 activation have been associated with the development of a tumorigenic phenotype in several cancers [1], [16]–[24]. Hence, the STAT3 pathway is a popular target for chemotherapeutic agents.

RKIP is a member of the phosphatidylethanolamine-binding protein family. In contrast to STAT3, RKIP antagonizes multiple cell-survival pathways, including the Ras-Raf-1 pathway [25], NF-κB (Nuclear Factor kappa Beta) [26], and GRK2 (G Protein-Coupled Receptor Kinase 2) [27] and activates others, like GSK3β [28]. RKIP is required for some human cancer cells to undergo drug-induced apoptosis [29]. RKIP is a metastasis suppressor in colon, breast, melanoma and prostate cancer and its expression is predictive of clinical outcome: better outcome with higher expression [30]–[35]. In addition, there is an inverse relationship between clinical outcome for gastric cancer patients and expression of RKIP and STAT3 [36]. RKIP expression levels vary in prostate and breast cancer cell lines depending on their metastatic capacity; as the levels of RKIP expression decreases, metastatic-potential of the cancer increases [37]. The lower levels of RKIP in these cells are caused by the direct inhibition of RKIP transcription by the zinc-transcriptional repressor protein Snail [37], which has also been found to down-regulate the tumor metastasis suppressor protein E-cadherin [38].

The article "Raf Kinase Inhibitor Protein (RKIP) Blocks Signal Transducer and Activator of Transcription 3 (STAT3) Activation in Breast and Prostate Cancer" was retracted in 2021. Reasons: manipulated images; duplicated images; original data or images not available; unreliable data.

The anti-proliferative effects of microtubule inhibitors (MTIs), such as taxol, have been exploited for quite some time as potential chemotherapeutic agents preventing microvasculature proliferation and stimulating apoptosis of various tumor cell lines including breast and prostate cancer cells [39], [40]. 2-Methoxyestradiol (2-ME2) is an estrogen-derived mammalian metabolite that has antitumor and antiangiogenic effects [41]; it causes apoptosis by inhibiting oncogenic proteins such as HIF-1α and disrupting microtubule polymerization via weak competitive binding to colchicine-binding sites [42]. ENMD-1198, an analog of 2-ME2 designed to retain the same mechanisms of action as 2-ME2 without undergoing the rapid *in vivo* metabolism of 2-ME2, was tested in a Phase I clinical trial. Not only does ENMD-1198 inhibit HIF1-α, but it also decreases STAT3 and NF-κB levels [43]. MKC-1 is a cell-cycle inhibitor that prevents mitotic spindle formation by interacting at the colchicine-binding site of microtubules [44]. MKC-1 also antagonizes the Akt-mTOR signaling pathway, the most frequently mutated pathway in human tumors with mutations that promote tumor progression and decrease survival among cancer patients [45].

In this study we examined the role of RKIP in the apoptotic inducing effects of MTIs and whether RKIP modulates MTI-mediated STAT3 activation in multiple experimental models [43], [44]. Through our experiments, we gained additional understanding of the multifunctional role and mechanisms by which RKIP inhibits cell survival and promotes apoptosis.

## Materials and Methods

### Ethics Statement

The animal care facilities at Rhode Island Hospital operate in full compliance with the OLAW/PHS policy on the Humane Care and use of Laboratory Animals and the USDA Animal Welfare act. The Hospital's NIH Assurance number is A-3922-01 and the USDA Registration number is 15-R-002. This study was performed with approval from Rhode Island Hospital IAUCUC CMT #0169-08. Any animal that exhibited anorexia or decreased water intake for 24 hours or decreased activity, hunched posture, excessive grooming or any other overt sign of distress was euthanized to limit further suffering. A 15% reduction in body weight compared to cage mates was also considered significant and affected animals were euthanized by CO2 asphyxiation.

The article "Raf Kinase Inhibitor Protein (RKIP) Blocks Signal Transducer and Activator of Transcription 3 (STAT3) Activation in Breast and Prostate Cancer" was retracted in 2021. Reasons: manipulated images; duplicated images; original data or images not available; unreliable data.

### Materials

2-ME2, ENMD-1198 and MKC-1 were provided by Entremed (Rockville, MD). All reagents and chemicals were purchased from Sigma Chemical Co. (St. Louis, MO) unless otherwise noted. Protein quantification reagents were obtained from Bio-Rad Laboratories, Inc. (Hercules, CA). Enhanced chemiluminescence reagents and secondary mouse and rabbit horseradish peroxidase-conjugated antibodies for Western blot analysis were ordered from GE Healthcare (Arlington Heights, IL). The antibodies to Src pY^416^ (2101S), STAT3 pY^705^ (9131S) and PARP (9542S) were purchased from Cell Signaling Technology (Beverly, MA); the RKIP (07-137), VEGF (06-585), Muc1 (05-652) and Cxcr4 (PC389) were purchased from Millipore (Hopkington, MA); the actin-HRP (sc-1616), c-Src (sc-19) and STAT3 (sc-482) antibodies were purchased from Santa Cruz Biotechnology (Santa Cruz, CA).

### Cells and Plasmids

The human prostate carcinoma cell lines PC3 and DU145, human breast carcinoma MDA-MB231 (MDA) and human normal renal epithelial cell lines 293T cells were purchased from ATCC (Rockville, MD). The cell lines in our lab were used between passage numbers 35-45. The prostate and breast cancer cells were grown in RPMI 1640 medium and 293T cells were grown in Dulbecco's modified Eagles medium. All cell lines were supplemented with 10% fetal calf serum, glutamine, non-essential amino acids, 100 units/ml penicillin and 50 units/ml streptomycin and cultured in a humidified incubator at 37°C containing 5% CO_2_. The expression plasmids for pcDNA3 c-myc STAT3, HA-STAT3, CMV-HA-RKIP, CMV-FLAG-RKIP and c-Src have been described [6], [29].

For RNAi-based silencing of expression of RKIP in the MDA cells, we prepared knockdown cells expressing the small interfering RNAs (siRNAs) specific for human RKIP or a firefly luciferase-specific siRNA as control from the short hairpin RNA (shRNA) expression vectors pSUPER.retro-puro (Oligoengene). The target sequences were: 5′GATTCAGGGAAGCTCTACA-3′ (RKIP-1/PEBP-1) and 5′ CGTACGCGGAATACTTCGA-3′ (firefly luciferase control). RKIP was over expressed in MDA cells by retroviral-mediated gene transfer. Retroviral constructs encoding N-terminally FLAG-tagged rat RKIP in the pQCXIP (Clontech) vector were used to generate RKIP-over expressing MDA cells as previously described [29]. Expression of the tagged RKIP fusions was confirmed by Western blot analysis.

### Cell Transfection

Cells were transiently transfected using the Lipofectamine transfection reagent (Invitrogen) according to the manufacturer's protocol. Transfection conditions were assessed and optimized by FACS analysis of cells transfected with a Green Fluorescent Protein (GFP)-expressing plasmid. Transfection efficiencies were consistently high (approximately 88–93% of cells). Total DNA quantities between 1 and 3 μg were transfected per sample.

The article "Raf Kinase Inhibitor Protein (RKIP) Blocks Signal Transducer and Activator of Transcription 3 (STAT3) Activation in Breast and Prostate Cancer" was retracted in 2021. Reasons: manipulated images; duplicated images; original data or images not available; unreliable data.

### Western Blot Analysis

Total cell extracts were prepared as previously described [46]. Protein concentrations of lysates were determined using the Bradford assay kit (BioRad). Proteins were separated by SDS-PAGE and electrophoretically transferred from the gel to nitrocellulose membranes (GE Healthcare). Proteins recognized by the antibodies were detected by enhanced chemilluminescence reagents (GE Healthcare). Densitometry of Western blots were performed according to the protocol listed at the following site: http://lukemiller.org/journal/2007/. Actin was used for normalization of loading of protein, and band densities were determined using Photoshop CS6. The relative intensity was determined by dividing the absolute intensity of each sample band by the absolute intensity of the Actin loading control.

### Flow Cytometry Analysis

The percentage of apoptotic cells (sub-G_O_) was determined by flow cytometric analysis of propidium iodide stained cells. The analysis was performed using a dual laser FACSCalibur flow cytometer (Becton Dickinson) with cell cycle modeling and analysis software from Modfit LT (Verity Software House, Inc., Topsham, MN) as previously described [46]. All experiments were repeated at least 3 times.

### Luciferase Reporter Assay

Cells (5 × 10^5^ cells/60 mm dish) were transiently transfected with 0.5 μg of a reporter plasmid containing STAT3 binding SIE-fragment of the promoter region of mouse IRF1 gene (p2xSIE-Luc) or the RKIP promoter using lipofectamine in serum-free medium [6], [37]. After 4 h OptiMEM, containing 20% FBS (final concentration), was added to the cells. To normalize transfection efficiencies, approximately 12 h after batch transfection of tissue culture dishes with the appropriate plasmids, cells were trypsinized, harvested and re-seeded into the appropriate number of dishes required for the individual experiment. After 12 h the cells were left untreated or treated with the indicated drug for the indicated time. Cells were harvested by scrapping, washing twice with PBS and lysing in passive lysis buffer (Promega, Madison, WI). The luciferase activity in the cytosolic supernatant was evaluated using the Dual Luciferase Reporter Assay (Promega) and measured using a luminometer to estimate transcriptional activity.

### Application of Small Interfering RNA (siRNA) against RKIP

DU145 cells were plated in a 6-well plate 24 h prior to transfection in an antibiotic-free growth medium. RKIP siRNA (Santa Cruz Biotechnology Inc.), or a relevant amount of a control siRNA solution was mixed with transfection reagent in OptiMEM. Complex formation was allowed for 30 min at room temperature. The mix was added to OptiMEM-washed cells together with OptiMEM and incubated for 6 h. At 6 h 1 ml of medium supplemented with 20% FBS was added to the cells and incubation was continued for a total of 48 h before treatment and cell harvesting. RKIP inhibition at the protein level was confirmed using Western blot analysis.

The article "Raf Kinase Inhibitor Protein (RKIP) Blocks Signal Transducer and Activator of Transcription 3 (STAT3) Activation in Breast and Prostate Cancer" was retracted in 2021. Reasons: manipulated images; duplicated images; original data or images not available; unreliable data.

### Electrophoretic Gel Mobility Shift Assays (EMSA)

Cells (10^6^) transfected with EV and HA-RKIP then treated with 40 ng/ml IL-6 for 12 h were harvested after treatment and washed twice with cold Dulbecco's PBS (Cellgro). After washing, the cells were lysed in 1 ml of NP40 lysis buffer (10 mM Tris-HCl pH 7.4, 10 mM NaCl, 3 mM MgCl_2_, 0.5% NP40 and 0.1 mM EDTA) on ice for 5 min. Samples were centrifuged at 300 × g at 4°C for 5 min. The pellet was washed twice in NP40 buffer. Nuclei were then lysed in nuclear extraction buffer (20 mM HEPES pH 7.9, 25% glycerol, 0.42 mM NaCl, 1.5 mM MgCl_2_, 0.2 mM EDTA, 0.5 mM phenylmethylsulfonyl fluoride, and 0.5 mM DTT) and sonicated for 10 s at 4°C. The protein concentration was determined using the Bio-Rad protein assay. The nuclear proteins were frozen at −80°C. Both buffers contained the complete protease inhibitor cocktail tablets from Roche. Nuclear protein (10 μg) was mixed for 30 min at room temperature with Biotin-labeled oligonucleotide probe STAT3, using the EMSA Kit purchased from Panomics™ (Panomics, Inc. Redwood City CA), following the manufacturer's instructions. 10 μl was subjected to denaturing 5% polyacrylamide gel electrophoresis and transferred to Nylon transfer membrane Hybond-N+ (Amersham) using the Trans-Blot® SD semi-dry Transfer cell System (Bio-Rad). The membranes were transferred to a UV Cross-linker FB-UVXL-1000 Fisher technology (Fisher Scientific) for 3 min. The detection was made as per the manufacturer's instructions, after the membranes were exposed using Hyperfilm ECL (GE Healthcare). The oligonucleotide sequences used for STAT 3 were: 5′-GATCCTTCTGGGAATTCC TAGATC-3′ as described [18], [47].

### STAT3-DNA Binding

A standard transcription factor enrichment assay was modified to assess STAT3 dimer binding to DNA. MDA cells were transiently transfected with an empty vector or an expression plasmid for RKIP. After 48 h, some cells were treated with IL-6 (40 ng/ml) for 12 h. Cells were harvested, and cell lysates were generated as previously described [18]. Four mg of total protein/condition was incubated overnight at 4°C in 3 ml of 100 mM HEPES-KOH (pH 7.9), 25 mM MgCl_2_, 300 mM KCl, 50 mM dithiothreitol, 0.5% Nonidet P-40, and 50% glycerol, containing 50 μg of the STAT3-DNA binding site oligonucleotide (5'-GATCCTTCTGGGAATTCCTAGATC-3') [47] agarose conjugate. Agarose beads were then removed by centrifugation, washed, and incubated in 50 μl of Laemmli buffer for 10 min at 100°C. Samples were then analyzed by Western blot analysis for STAT3 content.

The article "Raf Kinase Inhibitor Protein (RKIP) Blocks Signal Transducer and Activator of Transcription 3 (STAT3) Activation in Breast and Prostate Cancer" was retracted in 2021. Reasons: manipulated images; duplicated images; original data or images not available; unreliable data.

### Immunoprecipitation Assay

Cells were transfected with EV or the indicated plasmids for 48 h. In the experiment investigating IL-6 stimulation, cells were treated with 40 ng/ml IL-6 for 2 h. The cells were lysed in RIPA buffer. Five percent of the sample was removed to verify and analyze proteins present for the immunoprecipitation input. Approximately 1.5 mg of protein was incubated with 3 μg of monoclonal c-Myc antibody for 4 hr at 4°C. Immunocomplexes were collected on protein G-agarose beads separated 10% SDS-PAGE and electroblotted to nitrocellulose membrane. Proteins were detected after incubation with specific antibodies described and identified using the ECL detection system.

### Identification of Proteins Interacting with RKIP via Liquid Chromatography-Mass Spectrometry (LC-MS/MS)

Cells were transfected with HA-RKIP for 48 h. Lysed cells were immunoprecipitated with an antibody to HA and proteins were separated via 10% SDS-PAGE. The gel was stained with coomasie and the gel bands were excised by extracting gel particles with glass Pasteur pipettes. Sample preparation, including protein alkylation before proteolytic digestion, was performed as previously described [48]. After alkylation, the solution was removed and the gel pieces washed and dried. After rehydratation for 15 minutes at 4°C in digestion buffer consisting of 0.05 M ammonium bicarbonate, 5 mM CaCl_2_ and 12.5 μg/mL trypsin (porcine, sequence grade, Promega, Madison, WI, USA), the proteins were digested. After allowing the gel plugs to swell for 15 minutes, an additional volume of digestion buffer was added to cover the gel plugs that had completely adsorbed all initially added buffer, and the samples were then placed for 16 h in an incubator set at 37°C. After digestion, the peptides were recovered from the mixture by centrifugation (Eppendorf centrifuge). Peptides remaining in the gel were extracted with a solution of 50% (v/v) acetonitrile containing 1% (v/v) TFA (Pierce) in 25 mM ammonium bicarbonate for 10 min with shaking and subsequently pooled with the first fraction. The tryptic digest was held at −80°C until ready for LC-MS/MS analysis.

Tryptic “in-gel” or “in-solution” digests were separated with an RP column (C-18 PepMap 100, LC Packings/Dionex, Sunnyvale, CA, USA) [49]. The gradient was starting with 5% (v/v) acetonitrile in 0.1% (v/v) formic acid to 35% acetonitrile in formic acid (solvent B) for 75 minutes. The column eluate was introduced directly onto a QSTAR XL mass spectrometer (SCIEX and Applied Biosystems, Concord, Ontario, Canada) via ESI. Candidate ion selection, fragmentation and data collection were performed as described previously [50]. Protein identifications were performed with ProteinPilot software (Sciex and Applied Biosystems), using a human “RefSeq” databases from NCBI (http://www.ncbi.nim.nih.gov/RefSeq/). This software is the successor of ProID and ProGroup, and uses the same scoring method. Briefly, given a protein score S, the likelihood that the protein assignment is incorrect is 10^-S^, and the scores above *2.0* require that at least two sequence-independent peptides be identified. Protein identification was performed in at least two independent experiments.

The article "Raf Kinase Inhibitor Protein (RKIP) Blocks Signal Transducer and Activator of Transcription 3 (STAT3) Activation in Breast and Prostate Cancer" was retracted in 2021. Reasons: manipulated images; duplicated images; original data or images not available; unreliable data.

### Wound Healing/Scratch Assay

MDA MB-231 cells were seeded in 60 mm dishes containing glass coverslips at a density of 2×10^5^ cells/dish in RPMI 1640 medium containing 10% FBS [51] The cells were transiently transfected the following day with the indicated plasmids (see results). The confluent cells (∼85%) were starved in starvation medium for 18 h. and a wound line was drawn across the adherent cells on the glass coverslip. Non adherent cells were removed by washing the dishes with PBS. The cells were incubated in medium containing 1% FBS and after an additional 24 h, the cells were washed, fixed and stained with crystal violet and the cells migrating into the wound space counted.

### Growth of Tumor Xenografts

MDA cells (10^7^) that stably express: 1). empty vector, 2). activated and over expressed STAT3, 3). over expressed RKIP, 4). RKIP knockout and 5). activated and over expressed STAT3 and over expressed RKIP were injected into the two rear dorsal flanks of 6 week old female NU/J mice (Jackson Labs). After tumor implantation, mice were weighed and had tumor measurements taken twice weekly, starting on day 1. These tumor measurements were converted to tumor weight (mg) using an established formula: Weight (mg)  =  length × width (mm^2^)/2. Experiments were terminated when tumors in control animals reached a size of approximately 0.5 g. At termination, all of the mice were weighed and sacrificed, and their tumors excised.

### Statistical methods

All cell culture experiments were repeated at least 3 times, unless indicated otherwise, and paired t-tests were performed to determine statistical significance.

## Results

### 

#### RKIP over expression results in the reduction of c-Src-mediated STAT3 activation

C-Src-triggered STAT3 activation enhances breast cancer progression and prevents depolymerization of microtubules [15], [52]. Phosphorylated STAT3 participates in c-Src- and cytokine-mediated signal transduction [53]. Therefore, to explore the role of RKIP on c-Src-mediated STAT3 activation, MDA cells were transiently transfected with c-Src, RKIP, or the combination in the presence or absence of ENMD.

The article "Raf Kinase Inhibitor Protein (RKIP) Blocks Signal Transducer and Activator of Transcription 3 (STAT3) Activation in Breast and Prostate Cancer" was retracted in 2021. Reasons: manipulated images; duplicated images; original data or images not available; unreliable data.

Our results indicate a 2.9 fold increase (relative intensity 0.41 vs. 1.3) of STAT3 pY^705^ phosphorylation after transient transfection with c-Src when compared to untreated empty vector cells (Fig. 1A). In cells transiently transfected with c-Src *and*: a) co-transfected with HA-RKIP, STAT3 pY^705^ phosphorylation was reduced 38% (relative intensity 1.3 vs. 0.81); b) treated with ENMD treatment of c-Src transfected cells lowered STAT3 pY^705^ phosphorylation 43% (relative intensity 1.3 vs. 0.74); and c) co-transfected with HA-RKIP and treated with ENMD, STAT3 pY^705^ phosphorylation was reduced 47% (relative intensity 1.3 vs. 0.7).

**Figure 1:** ENMD-1198 inhibits c-Src-mediated STAT3 activation. (A)MDA-231 cells were transiently transfected with expression plasmids for c-Src and HA-RKIP for 48 h. Following this, the cells were treated with ENMD-1198 for 24 h and samples prepared for Western blot analysis and examined for the indicated proteins. Densitometry was performed and the relative intensity when compared to Actin for lanes 1-8, respectively, were: RKIP (top band): 0.225, 0.32, 0.81, 0.22, 0.85, 0.22, 1.02, 0.76; RKIP (bottom band): 0.42, 0.5, 0.4, 0.73, 0.4, 0.59, 0.68, 0.6; STAT3 pY^705^: 0.41, 1.3, 0.31, 0.10, 0.81, 0.74, 0.20, 0.70; STAT3: 0.075, 0.048, 0.059, 0.049, 0.042, 0.044, 0.033, 0.071; c-Src pY^416^: 0.22, 1.15, 0.59, 0.34, 0.75, 0.72, 0.16, 0.29; c-Src: 0.24, 0.37, 0.24, 0.31, 0.55, 0.31, 0.49, 0.5. (B) A STAT3 luciferase reporter assay was performed under the experimental conditions described in *A*. Cells were transiently transfected with a luciferase plasmid containing the consensus DNA STAT3 binding sequence for the SIE fragment of the promoter region of mouse *IRF1* gene for 48 h. Some cells were treated with ENMD-1198 for an additional 24 h. Luciferase activity was measured in cytosol extracts and compared with activity observed in non-treated (control) cells, in which the observed activity was set at arbitrary units. A paired t-test was performed to analyze the increase or decrease in STAT3 reporter activity: *(p<0.00000001) in c-Src transfected cells when compared to the empty vector; **(p<0.00000005) decrease in transcriptional activity in cells transfected with c-Src and RKIP and ***(p<0.00005) in cells transfected with c-Src and treated with ENMD-1198 and ****(p<0.000005) in cells transfected with c-Src, RKIP and treated with ENMD-1198, when compared to c-Src. EV = empty vector. (*bars*  =  mean ± S.D., of 2 experiments performed in triplicate). (C) Top, Western blot analysis was performed in cells transiently transfected with RKIP or EV for 48 h. Some cells were treated for 2 h with 40 ng/ml IL-6, whole cell extracts prepared and analyzed for the expression of the indicated proteins. Densitometry was performed and the relative intensity when compared to Actin for lanes 1-4, respectively were: STAT3 pY^705^: 0.64, 2.82, 1.3, 1.4; STAT3: 1.1, 1.2, 1.8, 1.3. Bottom, STAT3 luciferase assay was performed in MDA cells transiently transfected with STAT3 luciferase reporter construct or an expression vector for RKIP. After 48 h, some of the cells were treated with 40 ng/ml of IL-6 for 6 h. Cells were harvested and luciferase reporter activity measured. A paired t-test was performed demonstrating the increase in transcriptional activity of cells treated with *(p<0.000003) IL-6 when compared to EV. A decrease in transcriptional activity was observed in cells **(p<0.00004) transfected with RKIP and treated with IL-6 when compared to cells treated with IL-6 (*bars*  =  mean ± S.D., of 2 experiments performed in triplicate). (D) The same experiment was performed in DU145 prostate cancer cells as described in (C). Top: Western blot analysis of the inhibition of IL-6-mediated STAT3 phosphorylation by RKIP overexpression under the same experimental conditions described in (C). Densitometry was performed and the relative intensity (fold increase) when compared to Actin for lanes 1–4, respectively were: STAT3 pY^705^: 022, 0.78, 0.24, 0.18; STAT3: 0.75, 0.61, 1.3, 0.67. Bottom: STAT3 luciferase assay was performed in DU145 cells transiently transfected with STAT3 luciferase reporter construct or an expression vector for RKIP. A paired t-test was performed demonstrating the increase in transcriptional activity of cells treated with *(p<0.0004) IL-6 when compared to EV. A decrease in transcriptional activity was observed in cells **(p<0.0002) transfected with RKIP and treated with IL-6 when compared to cells treated with IL-6 (*bars*  =  mean ± S.D., of 2 experiments performed in triplicate). (E) STAT3 DNA binding activity was examined using the STAT3 EMSA kit purchased from Panamoics according to the manufacturer's instructions. Cells (10^6^) were transfected with EV or RKIP for 48 h. Some cells were treated with 40 ng/ml IL-6 for 6 h. Cells were harvested, washed and lysed in NP-40 lysis buffer. Nuclei were isolated and lysed according to the manufacturer's instructions. Nuclear protein (10 μg) was mixed for 30 min at room temperature with Biotin-labeled oligonucleotide probe STAT3, using the Panaomics EMSA Kit. The detection was made as per the manufactory's instructions. (F) Western blot analysis of STAT3-DNA binding as a function of RKIP overexpression and IL-6 treatment was determined. Cell lysates were generated, particulate material then was removed by centrifugation, and the resulting supernatant (1.5 mg of total protein/condition) was incubated overnight at 4°C in binding buffer containing 50 μg of STAT3-DNA binding site oligonucleotide-agarose conjugate. The resulting supernatant was analyzed by Western blot methods to assess STAT3 content [18].

The article "Raf Kinase Inhibitor Protein (RKIP) Blocks Signal Transducer and Activator of Transcription 3 (STAT3) Activation in Breast and Prostate Cancer" was retracted in 2021. Reasons: manipulated images; duplicated images; original data or images not available; unreliable data.

C-Src transient transfection results indicate a 5.3 fold increase (relative intensity 0.22 vs. 1.15) of c-Src pY^416^ phosphorylation when compared to empty vector transfected MDA cells (Fig. 1A). In cells transiently transfected with c-Src *and*: a) co-transfected with HA-RKIP, c-Src pY^416^ phosphorylation was reduced 34% (relative intensity 1.15 vs. 0.75); b) treated with ENMD, c-Src pY^416^ phosphorylation was reduced 40% (relative intensity 1.15 vs. 0.72); and c) co-transfected with HA-RKIP and treated with ENMD, c-Src pY^416^ phosphorylation was reduced 70% (relative intensity 1.15 vs. 0.29). Collectively these results indicate that HA-RKIP overexpression and ENMD treatment can, independently and concomitantly, inhibit c-Src-mediated STAT3 pY^705^ and c-Src pY^416^ phosphorylation.

The results of the Western blot analysis were confirmed by a luciferase reporter assay in MDA cells. MDA cells were transiently transfected with a reporter plasmid containing a STAT3-binding SIE-fragment of the promoter region of mouse IRF1 gene (p2xSIE-Luc) in serum-free medium [6]. Transient transfection of MDA cells with c-Src resulted in a significant (7-fold) increase in STAT3 luciferase reporter activity (p<0.00000001) when compared to the empty vector control (Fig. 1B). There was a greater than 4-fold (p<0.00000005) decrease in transcriptional activity in cells transfected with c-Src and RKIP when compared to c-Src alone (Fig. 1B).

### RKIP over expression results in the reduction of IL-6-mediated STAT3 activation

To determine if the inhibition of STAT3 phosphorylation and transcriptional activation by RKIP was only c-Src-specific, we examined the ability of RKIP to inhibit IL-6-mediated STAT3 activation. MDA cells were transiently transfected with CMV empty vector or HA-RKIP for 24 h and then treated with IL-6 (40 ng/ml) for 2 h. As shown in Figure 1C, treatment of CMV empty vector-transfected cells with IL-6 resulted in significant STAT3 pY^705^ transcriptional activation, as measured by a STAT3 luciferase reporter assay (p<0.000003). Transient transfection of HA-RKIP inhibited STAT3 phosphorylation and IL-6 mediated transcriptional activation (p<0.00004) (Fig. 1C).

The article "Raf Kinase Inhibitor Protein (RKIP) Blocks Signal Transducer and Activator of Transcription 3 (STAT3) Activation in Breast and Prostate Cancer" was retracted in 2021. Reasons: manipulated images; duplicated images; original data or images not available; unreliable data.

In MDA cells treated with IL-6, we observed a 3.5-fold increase (relative intensity 0.64 vs. 2.82) of STAT3 pY^705^ phosphorylation (Fig. 1C). Transient transfection of HA-RKIP inhibited IL-6 mediated STAT3 pY^705^ phosphorylation 50% (relative intensity 2.82 vs. 1.4). These results demonstrate that HA-RKIP is a potent inhibitor of IL-6-mediated STAT3 pY^705^ phosphorylation.

To determine if the inhibition of STAT3 phosphorylation and transcriptional activation was specific to breast cancer cells, we performed the same experiment described in Figure 1C, with DU145 prostate cancer cells. Our results indicate that transfection of RKIP inhibited IL-6-mediated STAT3 transcriptional activation (p<0.0002) and a 76% inhibition of STAT3 pY^705^ phosphorylation (relative intensity 0.78 vs. 0.18) (Fig. 1D). These results demonstrate that RKIP can also inhibit IL-6-mediated STAT3 activation and phosphorylation in prostate cancer cells.

We examined the ability of RKIP to inhibit IL-6-dependent STAT3 DNA binding. Extracts were generated from cells transfected with RKIP or EV for 48 h and then exposed for 12 h to 40 ng/ml IL-6. In initial experiments, STAT3 binding to DNA was assessed by an electrophoretic mobility shift assay (EMSA) using the Panomics STAT3 EMSA kit. Assessment of STAT3 DNA binding by EMSA revealed that IL-6 promoted STAT3 DNA binding, the level of which was significantly reduced by RKIP over expression. The results of this analysis revealed that IL-6 promoted STAT3 DNA binding. The consequence of this reduction in the cellular content of STAT3 pY^705^ by RKIP over expression was a significant reduction in STAT3 dimer binding to DNA (Fig. 1E). To confirm the specificity of this effect, STAT3 binding to DNA also was assessed in total cell extracts by exposure to the STAT3 DNA binding site consensus sequence immobilized on agarose beads. Western blot analysis revealed an increase in binding after IL-6 treatment and again a dramatic reduction in STAT3 dimer recovery in cells transfected with RKIP (Fig. 1F). These results suggest that one mechanism of RKIP-mediated inhibition of STAT3 activation occurs by preventing STAT3 DNA binding via inhibition of phosphorylation.

### MTIs induce RKIP expression in a prostate cancer cell line

Microtubule inhibitors such as taxol are important agents that have been used extensively and investigated for the treatment of breast and prostate cancer for many years [54]-[56]. We hypothesized that the anti-tumor effects of MTIs are not only mediated by a direct effect on microtubules, but also by the induction of tumor suppressor RKIP. Many naturally occurring or synthetic compounds are known to induce the expression of RKIP [57]. Human prostate and breast carcinoma cells undergo apoptosis when treated with various chemotherapeutic compounds, including camptothecins (CPT) [46] cisplatin [58] and taxol [39], [40] In addition, we have shown that RKIP is required for chemotherapy-triggered apoptosis [29].

The article "Raf Kinase Inhibitor Protein (RKIP) Blocks Signal Transducer and Activator of Transcription 3 (STAT3) Activation in Breast and Prostate Cancer" was retracted in 2021. Reasons: manipulated images; duplicated images; original data or images not available; unreliable data.

Therefore, we investigated the effects of MTIs on prostate and breast cancer cell apoptosis and RKIP protein expression. DU145, PC3 and MDA cells were treated with ENMD-1198 and MKC-1 at IC_50_ concentration (200 nM) for 6 or 12 h and were then analyzed via Western blot analysis. As shown in Fig. 2A, both MTIs induced the expression of RKIP in DU145 but not PC3 cells or MDA cells. We examined the time course for RKIP induction in DU145 cells. EMND-1198-treated DU145 cells showed a more rapid increase of RKIP expression when compared to cells treated with MKC-1 (Fig. 2B).

**Figure 2:** Microtubule inhibitors cause cell cycle arrest and induce RKIP expression. (A) DU145 and PC3 cells were treated with ENMD-1198 or MKC-1. Cells were harvested and washed twice with PBS and whole cell lysates were prepared for Western blot analysis as we have previously reported [28]. Proteins (unless indicated 50 μg/sample was used for Western blot analysis) were separated by 10% SDS-PAGE, transferred to nitrocellulose and analyzed with antibodies to the indicated proteins. *Note: for all Western blots described in this Figure legend and for all other subsequent Figure legends, the exposure time used to identify the various proteins was variable*. (B) DU145 cells were treated with 200 nM ENMD-1198 or MKC-1 for 6 or 12 h. Cells were prepared for Western blot analysis for the indicated proteins. (C) DU145, PC3 prostate and MDA breast cancer cells (1 × 10^5^) were used for FACS analysis after treatment with the indicated concentrations of ENMD-1198 or MKC-1. Cells were harvested, washed twice with phosphate buffered saline (PBS) and prepared for flow cytometry as previously described (43). Analysis for apoptosis was performed using a FACSCalibur flow cytometer (Data represents the mean ± S.D., of 2 independent experiments performed in duplicate). (D) (Left panel) PC3 and MDA cells were transiently transfected with HA-RKIP expression plasmid for 48 h. Whole cell lysates were prepared and Western blot analysis was performed as described in A for the indicated proteins. *Note for this and all other subsequent experiments described where RKIP was transfected into cells, the lower RKIP band represents endogenous RKIP, while the upper RKIP band represents ectopic RKIP (HA-RKIP)*. (Right panel), DU145 cells were treated with ENMD-1198 or MKC-1 for 24 h. Whole cell lysates were prepared and Western blot analysis was performed for the indicated proteins. (E, top) DU145 cells were transiently transfected with various combinations with expression plasmids for RKIP, RKIP siRNA, scramble siRNA or empty vector (EV) for 48 h. The cells were treated with 200 nM ENMD-1198 for 24 h. Cells were harvested and analyzed for apoptosis as described in (C). A paired t-test was performed to analyze the increase in apoptosis in cells when compared to empty vector (EV): *(p<0.001) transiently transfected with RKIP; **(p<0.00007) treated with ENMD-1198; ***(p<0.0002) with the combination of RKIP transfection and ENMD-1198 treatment. Scrmbl = scrambled siRNA. A decrease in apoptosis was observed ****(p<0.000012) in cells treated with ENMD-1198 when compared to cells transiently transfected with RKIP siRNA and treated with ENMD-1198. (Data represents the mean ± S.D., of 2 independent experiments performed in triplicate). (E, bottom) Western blot analysis of the same experimental conditions described in Fig. 2E, top. The Western blot analysis was repeated 3 times and the Figure is representative of one of the experiments. Densitometry was performed and the relative intensity (fold increase) when compared to Actin for lanes 1-8, respectively were 0.78, 1.7, 0.19, 0.84, 0.99, 0.67, 0.36 and 0.92.

The article "Raf Kinase Inhibitor Protein (RKIP) Blocks Signal Transducer and Activator of Transcription 3 (STAT3) Activation in Breast and Prostate Cancer" was retracted in 2021. Reasons: manipulated images; duplicated images; original data or images not available; unreliable data.

### RKIP overexpression restores sensitivity to MTI-associated apoptosis in resistant cancer cells

We determined the apoptotic effects of MTIs in prostate and breast cancer cell lines using flow cytometry analysis. Cells were treated with ENMD-1198 or MKC-1 at the indicated concentrations for 24 h and were then collected and analyzed for apoptosis via flow cytometry (Fig. 2C). We found that the percentage of apoptosis substantially increased in a dose-dependent manner in DU145 prostate cancer cell lines treated with ENMD-1198 and MKC-1 (Fig. 2C). However, PC3 prostate and MDA breast cancer cells were resistant to MTI-induced apoptosis, (Fig. 2C). These results suggest that the resistance of PC3 and MDA cells to MTI-mediated apoptosis may be due to the lack of RKIP induction.

RKIP over expression sensitizes breast and prostate cancer cells to drug-induced apoptosis [35]. Therefore, we sought to determine whether over expression of RKIP could sensitize ENMD-1198-resistant PC3 prostate and MDA breast cancer cells to apoptosis. Both cell lines were transiently transfected with HA-RKIP expression plasmid for 24 h and were then treated with ENMD-1198 for 12 h. Our results indicate that MDA and PC3 cells underwent substantial cell death, as measured by Poly (ADP-ribose) polymerase (PARP) cleavage upon transfection with RKIP and treatment with ENMD-1198 (Fig. 2D). These results were reproduced in both cell lines after treatment with MKC-1 (data not shown). We also measured PARP cleavage upon treatment with ENMD-1198 and MKC-1 in DU145 cells. Both MTIs induced RKIP expression and PARP cleavage, as shown in Fig. 2D, right panel.

The article "Raf Kinase Inhibitor Protein (RKIP) Blocks Signal Transducer and Activator of Transcription 3 (STAT3) Activation in Breast and Prostate Cancer" was retracted in 2021. Reasons: manipulated images; duplicated images; original data or images not available; unreliable data.

To confirm that RKIP is required during MTI-triggered apoptosis, DU145 cells were transiently transfected with RKIP expression plasmid, RKIP siRNA, or scramble siRNA for 48 h and then treated with ENMD-1198 for 24 h. Our results indicate that there was a greater than 3-fold increase in apoptosis in DU145 cells transiently transfected with RKIP (p<0.001) or treated with ENMD-1198 (p<0.00007) and greater than 5-fold with the combination (p<0.0002) (Fig. 2D). In the presence of RKIP siRNA, apoptosis due to ENMD-1198 treatment was reduced greater than 3.5-fold (p<0.000012) when compared to the combination of RKIP transfection and ENMD-1198 treatment (Fig. 2E, top). The results from the siRNA experiment were substantiated by Western blot analysis (Fig. 2E, bottom). The expression of RKIP was reduced greater than 50% in cells transfected with RKIP siRNA (Fig. 2E, bottom). Collectively, our results indicate that the increase in endogenous RKIP is required for enhanced MTI-triggered apoptosis.

### RKIP inhibits JAK- and Raf-mediated STAT3 activation

Having determined that RKIP and ENMD-1198 were effective in inhibiting STAT3 activation and phosphorylation, we next focused on the ability of RKIP and ENMD-1198 to inhibit JAK-mediated activation of STAT3 using the luciferase reporter assay. We chose to use 293T renal epithelial cells to gain further understanding of RKIP function for three main reasons. First, it has been previously established that STAT3 is activated in DU145 and PC3 cells by more than one JAK kinase [59]. Second, we have previously shown that STAT3 expression was not changed by modulating RKIP expression in 293T cells [60] and third, because 293T cells have a higher transfection efficiency with the plasmids we were using, especially under the serum free conditions used in the experiments described below. 293T cells were transfected with the IRF-1 plasmid along with cDNA encoding either JAK1, 2, or 3 or TYK2 in the presence or absence of ENMD-1198 or transiently expressed HA-RKIP. Our data demonstrate that JAK1, 2, 3 and TYK2 were able to significantly stimulate STAT3 luciferase reporter activity (Fig. 3A). Ectopic RKIP expression significantly inhibited STAT3 luciferase reporter activity in cells transfected with JAK1 and 2, but not JAK3 or TYK2 (Fig 3A). Treatment of IRF-1 and JAK1, 2, 3 or TYK2 transfected cells with ENMD-1198 for 24 h did not affect STAT3 transcriptional reporter activity. The induction of RKIP occurs after 6 h of exposure to ENMD-1198 in some cell lines (Fig. 2B), which indicates that inhibition of JAK activity is ENMD-1198-independent. The inhibition of STAT3 luciferase reporter assay by HA-RKIP was comparable to the JAK inhibitors tyrphostin and AG490 (data not shown). We also examined the ability of RKIP to inhibit JAK1-, 2-mediated inhibition of STAT3 pY^705^ phosphorylation. Western blot analysis demonstrated that transiently expressed RKIP (0.5 μg) effectively inhibited JAK1- and 2-mediated phosphorylation of STAT3 (Fig. 3B).

The article "Raf Kinase Inhibitor Protein (RKIP) Blocks Signal Transducer and Activator of Transcription 3 (STAT3) Activation in Breast and Prostate Cancer" was retracted in 2021. Reasons: manipulated images; duplicated images; original data or images not available; unreliable data.

**Figure 3:** RKIP blocks JAK and Raf-mediated STAT3 activation. (A) RKIP inhibits JAK1, 2-triggered STAT3 activation. 293T cells were transfected with the Luc reporter construct containing 2× STAT3 binding SIE-fragment and co-transfected with either JAK1, 2, 3 or TYK2 in the presence or absence HA-RKIP and ENMD-1198. Cells were placed in serum free medium and cell extracts were subjected to luciferase assay to estimate transcriptional activity. Averages and standard deviations (error bars) of the values of luciferase activities from triplicates of 3 representative experiments are shown. (B) Western blot analysis demonstrating inhibition of STAT3 pY^705^ phosphorylation in HA-RKIP and JAK1 or 2 transiently transfected 293T cells. Raf-mediated STAT3 pY^705^ phosphorylation is inhibited by RKIP: (C) 293T cells were transfected with Raf-BXB, CMV empty vector or HA-RKIP. After 48 h cells were left untreated or exposed to IL-6 for 1 h. Cell lysates were analyzed by Western blot. (D) 293T cells were transfected with the STAT3 luciferase reporter construct and/or with EV, Raf-BXB or HA-RKIP. After 24 h, some cells were treated with PD98059 (PD) and after 48 h from the initial time of transfection, some cells were treated with IL-6 for 6 h. A paired t-test was performed indicating *(p<0.000005) increase in BXB transfected cells when compared to EV; decrease in STAT3 transcriptional activity **(p<0.00006) in PD treated cells transfected with BXB and ***(p<0.00004) in RKIP and BXB transfected cells when compared to the cells transfected with BXB. Luciferase reporter activities for triplicates of 3 representative experiments +/- s.d. are shown. Western blot analysis of cells transfected with the indicated proteins in the presence or absence of PD treatment.

RKIP was originally identified as an inhibitor of Raf [25], which is the activating kinase for the MAPK cascade. We examined the ability of Raf-BXB, an untagged constitutively active version of Raf [25], to phosphorylate STAT3 and the ability of RKIP to interfere with this process. Serum-starved 293T cells were transfected with Raf-BXB in the presence or absence of HA-RKIP expression vector. After 48 h in serum-free medium, cells were left untreated or exposed to 20 ng/ml of IL-6. As shown in Fig. 3C, Raf-BXB and IL-6 caused an increase in the STAT3 pY^705^ levels, an effect that appeared to be additive when cells were exposed to Raf-BXB and treated with IL-6 (Fig. 3C). This may be due to the fact that overexpression of BXB bypasses RKIP's constitutive role and leads to a regulatory loop that results in the phosphorylation of RKIP by ERK.

The article "Raf Kinase Inhibitor Protein (RKIP) Blocks Signal Transducer and Activator of Transcription 3 (STAT3) Activation in Breast and Prostate Cancer" was retracted in 2021. Reasons: manipulated images; duplicated images; original data or images not available; unreliable data.

Transient transfection with HA-RKIP blocked Raf-BXB and IL-6 STAT3 pY^705^ phosphorylation (Fig. 3C).

We investigated whether RKIP could block Raf-BXB-mediated-STAT3 activation as measured by a reporter plasmid containing STAT3-binding SIE-fragment transfected in 293T cells. Cells were transfected with Raf-BXB or HA-RKIP as described above and after 24 h were treated with the MAP-kinase inhibitor PD98059 for an additional 24 h. As shown in Fig. 3D, Raf-BXB caused significant (p<0.000005) induction of STAT3 transcriptional activity as measured by the luciferase reporter assay. Treatment with PD98059 for 24 h after transfection (p<0.00006) or transfection of 293T cells with HA-RKIP significantly (P<0.00004) inhibited Raf-BXB-mediated STAT3 activation (Fig. 3D). Interestingly, PD98059 reduces STAT3 pY705 in combination with BXB (data not shown). Our results indicate that RKIP can block Raf-dependent STAT3 pY^705^ phosphorylation and transcriptional activation. Our data also indicate that RKIP acts as a multiple kinase inhibitor as it inhibits JAK- and Raf-mediated STAT3 pY^705^ phosphorylation and transcriptional activation.

### RKIP interacts with, and inhibits STAT3 activation

To delineate the mechanism by which RKIP inhibits c-Src- and JAK1 and 2-mediated STAT3 activation, a series of RKIP deletion constructs (Fig. 4A, upper panel) were examined for their ability to inhibit JAK1-mediated STAT3 activation. As noted in Fig. 4A, middle panel, full-length and clone N60 RKIP expression constructs potently inhibited Src- and JAK1-mediated STAT3 phosphorylation. RKIP deletion constructs N93, C134 and C93 did not block c-Src-mediated STAT3 pY^705^ phosphorylation, shown with Western blot analysis (Fig. 4A, lower panel).

**Figure 4:** RKIP inhibits Src-STAT3 interaction. (A), top panel, Cartoon depicting a series of RKIP deletion constructs that were examined for their ability to inhibit c-Src- and JAK1-mediated STAT3 activation. *Middle panel*, Some of the deletion constructs were transfected in the presence of c-Src or JAK1 into cells for 48 h. Whole cell protein lysates were examined for the expression of STAT3, STAT3 pY^705^ and actin. *Lower panel*, Cells were transfected with EV, c-Src or RKIP deletion constructs N93 and C93. After 48 h, cells were harvested and whole cell lysates prepared to examine the expression of the indicated proteins via Western blot analysis. (B) Cells were transfected with c-myc EV, or the following tagged expression plasmids: myc-c-Src (2 μg), HA-STAT3 (2 μg), Flag-RKIP (4 μg) or the combination for 48 h. Cells were lysed in RIPA buffer, cellular debris removed, a portion of the sample removed as the IP input and the remaining supernatant incubated and rotated with an antibody to c-myc for 4 h at 4°C. Subsequently, protein G agarose was added and the samples rotated overnight at 4°C. Protein G agarose containing immuno complexes was extensively washed, 2× sample buffer added and the samples heated at 95°C for 5 min. Proteins were separated by SDS-PAGE, transferred onto nitrocellulose. The samples subjected to IP were divided in half. One filter was examined with an antibody to HA the other with an antibody to c-myc. The HA filter was stripped and examined for STAT3 levels. The input samples were examined for the expression of the indicated proteins. (C) Western blot analysis of cells transfected with EV (lane 1), c-Src (lane 2), HA-RKIP (lane 3) and c-Src + HA-RKIP (lane 4) to examine the expression of the indicated proteins that were separated on 15% SDS-PAGE. (D) RKIP inhibits c-Src-mediated MDA-231 cell migration. MDA-231 cells were transfected with empty vector, c-Src, c-, HA-RKIP, RKIP siRNA, scrambled siRNA or the combination. The cells were allowed to grow to near confluence. Cells were wounded with a pipette and after 24 h the migrated cells were fixed then stained with crystal violet and quantified. A paired t-test was performed indicating *(p<0.0002) an increase in migration in c-Src transfected MDA cells when compared to EV transfected cells and **(P<0.005) inhibition of c-Src-mediated increase in migration when compared to cells transfected with c-Src and RKIP. The data represents two independent experiments performed in triplicate.

The article "Raf Kinase Inhibitor Protein (RKIP) Blocks Signal Transducer and Activator of Transcription 3 (STAT3) Activation in Breast and Prostate Cancer" was retracted in 2021. Reasons: manipulated images; duplicated images; original data or images not available; unreliable data.

Although both N60 and C134 bind to Raf, clone N60 has a higher affinity than C134 for binding to Raf [29], suggesting that the N60 sequence may also have a greater ability to disrupt c-Src:STAT3 interactions. To determine whether there is any interaction among RKIP, c-Src, and STAT3, MDA cells were transiently transfected with the following series of epitope-tagged expression plasmids: c-myc empty vector, c-myc-Src and HA-STAT3, c-myc-Src and Flag-RKIP, HA-STAT3 and Flag-RKIP and c-myc-Src, HA-STAT3 and Flag-RKIP. We did not use the MDA RKIP stable cell line for this experiment because we did not have a stable cell line for c-Src. After 48 h, lysates were prepared and incubated with an antibody to c-myc as described in the Experimental Procedures section. Western blot analysis was performed and the nitrocellulose filter was analyzed by incubation to an antibody to HA. As shown in Fig. 4B, a constitutive interaction was noted between Src and STAT3. That interaction was no longer present in cells that were transfected with Src, STAT3, and RKIP. LC/MS was performed to determine if RKIP constitutively associated with c-Src, STAT3 or other proteins in the JAK/STAT pathway. Cells were transfected with HA-RKIP plasmid and cell lysates immunoprecipitated with an antibody to HA. After excision and “in gel” digestion the protein in one of the bands was identified as STAT3, the isoform 1 of signal transducer and activator of transcription 3 with a very high confidence (score 62.46). Thirty-four peptides belonging to this protein were identified, and the sequence coverage was 53.9%. This result supports our IP result indicating the interruption of Src:STAT3 association after RKIP over expression.

Activated Src (pY^416^) was observed in the Western blot analysis of the co-IP input samples transfected with c-myc, Src, and/or HA-STAT3. When Src was co-transfected with RKIP, however, Src was no longer in its activated phosphorylated form (Fig. 4B), indicating that RKIP inhibited Src autophosphorylation. These results further indicate the versatility of RKIP in blocking STAT3 activation.

We explored the consequence of RKIP disrupting Src-STAT3 interaction. Activated Src and STAT3 have been associated with promoting epithelial-mesenchymal transition (EMT) in tumor cells [61], [62]. We investigated the ability of RKIP over expression to inhibit c-Src-mediated induction of proteins that are intimately involved with EMT, migration, and angiogenesis. As shown in Fig. 4C, c-Src transient transfection of MDA cells resulted in the induction of Cxcr-4, VEGF and Muc1 protein expression, and RKIP over expression significantly inhibited the expression of these EMT-associated proteins (Figure 4C). To complement this result, we showed that transfection of MDA cells with c-Src resulted in an approximately 4-fold and significant increase (p<0.0002) in migration of MDA cells (Fig. 4D). In cells co-transfected with c-Src and RKIP, there was approximately a 60% reduction in migration (P<0.005) when compared to cells that had been transfected with c-Src (Fig. 4D). Transfection of MDA cells with RKIP siRNA did not effect Src-mediated migration. These results indicate that RKIP can inhibit c-Src-mediated MDA cell migration.

The article "Raf Kinase Inhibitor Protein (RKIP) Blocks Signal Transducer and Activator of Transcription 3 (STAT3) Activation in Breast and Prostate Cancer" was retracted in 2021. Reasons: manipulated images; duplicated images; original data or images not available; unreliable data.

### RKIP inhibits IL-6-mediated STAT3 activation in stably transfected cell lines

Our data thus far has indicated that RKIP can inhibit multiple mechanisms of STAT3 activation (Figs. 1, 3). Our experiments were performed with transient transfection over expression of RKIP (Figs. 1-3) and RKIP siRNA (Fig. 2). Therefore, to accurately assess the role of RKIP in the inhibition of STAT3 activation, stable MDA cell lines were created that over express (MDA RKIP) and do not express RKIP (knockdown, MDA si175). We examined the effect of IL-6 on STAT3 luciferase reporter activity in both models, including the appropriate empty vector controls. MDA EV and MDA RKIP were transfected with the STAT3 reporter and treated with IL-6 as previously described in Fig. 3. As shown in Fig. 5A, treatment of MDA EV cells with IL-6 resulted in a greater than 2.5 fold (p<0.007) increase in STAT3 luciferase reporter activity. In contrast, in MDA RKIP cells that stably over express RKIP there was a slight decrease (1-fold) in reporter activity when compared to untreated cells (Fig. 5A). In the knockdown cells, IL-6 treatment resulted in a greater than 2-fold increase in reporter activity in the MDA si175 empty vector control cells (Fig. 5B). In contrast, in the stable MDA si175 RKIP knockdown cells, IL-6 treatment resulted in a greater than 11-fold (p<0.005) increase in STAT3 luciferase reporter activity (Fig. 5B).

**Figure 5:** RKIP is required to inhibit STAT3 activation and breast tumor xenograft growth. (A) STAT3 luciferase reporter activity was performed as described in Figure 2 in cells treated with 40 ng/ml IL-6 for 6 h. *A*, represents MDA RKIP cells and (B) MDA si175 RKIP knockdown cells. Paired t-test was performed; *(p<0.007) in IL-6 treated cells when compared to EV control. Luciferase reporter activities for duplicate of 2 representative experiments +/- s.d. are shown. (C) Western blot analysis was performed in MDA RKIP and MDA si175 RKIP treated with 40 ng/ml IL-6 for 2 h. Whole cell lysates were examined for the expression of the indicated proteins. (D) MDA cells were implanted s.c. in the dorsal flanks of Nu/J female mice. Tumors were measured using calipers twice weekly, and volumes were calculated using the formula: weight (mg)  =  [width (mm)^2^ × length (mm)]/2. A paired t-test was performed indicating the decrease of RKIP *(p<0.002) or increase of **(p<0.008) si175RKIP, ***(p<0.002) STAT3 of tumor growth when compared to EV. A decrease in tumor growth was detected between STAT3 and RKIP/STAT3 ****(p<0.009). Mean tumor size for each treatment group is plotted (*n*  =  6) +/− s.d.

The article "Raf Kinase Inhibitor Protein (RKIP) Blocks Signal Transducer and Activator of Transcription 3 (STAT3) Activation in Breast and Prostate Cancer" was retracted in 2021. Reasons: manipulated images; duplicated images; original data or images not available; unreliable data.

We examined the effect of IL-6 treatment on STAT3 pY^705^ phosphorylation in MDA RKIP and MDA si175 cells. In MDA EV cells, IL-6 treatment resulted in STAT3 pY^705^ phosphorylation, but not in MDA RKIP cells (Fig. 5C). In contrast, in MDA si175 EV cells IL-6 treatment resulted in STAT3 pY^705^ phosphorylation, which was significantly increased in MDA si175 RKIP knockdown cells (Fig. 5C).

### RKIP blocks STAT3 promotion of tumor xenograft growth

STAT3 has been shown to promote breast cancer tumor growth [63], [64] and our results have shown that RKIP is a potent inhibitor of STAT3 activation *in vitro*. Therefore, we examined if RKIP could inhibit STAT3-mediated tumor xenograft growth. Our results indicate that mice inoculated with parental MDA EV cells had an average tumor growth of 215 mg (Fig. 5D). Mice inoculated with MDA RKIP had a 1.4-fold reduction in tumor mass (p<0.002), MDA si175 RKIP a 1.2-fold (p<0.008) and MDA STAT3 a 1.4-fold (p<0.002) increase in tumor mass when compared to MDA EV (Fig. 5D). MDA cells that over express RKIP and activated STAT3 had a 1.1-fold and not significant increase (p<0.13) in tumor growth when compared to MDA EV, but also a significant 1.3 fold (P<0.009) reduction in tumor mass when compared to MDA STAT3 (Fig. 5D). Taken together, our studies indicate that RKIP overexpression inhibits and RKIP ablation significantly enhances IL-6 mediated STAT3 activation and that RKIP can inhibit STAT3-mediated tumor growth. Our data suggest that RKIP is a native negative regulator of STAT3 activity.

## Discussion

In this study we show that MTIs ENMD-1198 and MKC-1 induced apoptosis in prostate and breast cancer cell lines is dependent upon the induction of RKIP. Src is able to induce and activate STAT3 expression and stabilize microtubules. MTIs inhibit STAT3 phosphorylation and in MTI-treated MDA breast cancer cells, where c-Src promotes STAT3 activation, we detected the inhibition of c-Src- and IL-6-mediated STAT3 phosphorylation and activation, effects that were greatly enhanced by RKIP over expression. IL-6-mediated STAT3 activation was RKIP dependent as demonstrated by the lack of STAT3 activation in MDA cells that over express RKIP and a significant enhancement of activation in cells that have knockdown of RKIP. In addition, RKIP blocked JAK1 and 2- and Raf-mediated STAT3 activation and STAT3-mediated tumor xenograft growth. Our studies demonstrate that RKIP: i) is required for MTI-mediated apoptosis; ii) inhibits JAK and Raf kinase activities; iii) inhibits Src association with STAT3 and iv) is required to inhibit STAT3 activation and STAT3-mediated tumor formation. Although over expression systems may be interpreted as artificial, our results with the knockdown of RKIP, or basically loss of RKIP function, indicate its pivotal role in STAT3 and c-Src activation, phosphorylation and tumor formation.

The article "Raf Kinase Inhibitor Protein (RKIP) Blocks Signal Transducer and Activator of Transcription 3 (STAT3) Activation in Breast and Prostate Cancer" was retracted in 2021. Reasons: manipulated images; duplicated images; original data or images not available; unreliable data.

Numerous chemotherapeutic agents act on the instability of MT polymerization to exert their cytotoxic effects, leading to cellular senescence, cell-cycle arrest, and apoptosis. For instance, taxane drugs such as Paclitaxel stabilize polymeric MTs in their GDP-bound state, preventing depolymerization [65]. MTIs like colchicine have the opposite effect: they bind to monomeric tubulin, preventing MT polymerization and thus causing polymerized MTs to destabilize and depolymerize. The MTIs used in this study bind to the colchicine-binding sites of tubulin inhibiting spindle formation, but also cause different downstream effects than original congeners, including the inhibition of the oncogene HIF1-α. Previous studies have shown the requirement of RKIP for chemotherapy-triggered apoptosis [29] and inhibition of metastasis in prostate cancer [31]. RKIP's role in mediating MT dynamics in prostate or breast cancer has not been given much emphasis despite recent findings implicating RKIP in the regulation of mitotic spindle checkpoints via association with centrosomes and kinetochores [66]. Specifically, RKIP induction activates Aurora B kinase, a spindle checkpoint regulator, via inhibition of Raf-1 [66]. RKIP also regulates MT dynamics by potently regulating STAT3 levels. Based on the results obtained in this study, we hypothesize that RKIP's ability to potentiate the apoptotic effects of the MTIs used in this study results from its multiple ways of regulating MT dynamics. It is has been suggested that MTIs indirectly cause MT instability by decreasing STAT3 levels. STAT3 inhibits the MT-destabilizing protein Stathmin, allowing MT polymerization to occur [15]. Therefore, identifying factors or compounds that negatively regulate MT polymerization-activators and further cause cell cycle arrest and apoptosis would be an important step in developing therapies. As we describe here, this can occur via RKIP over expression, which inhibits constitutive c-Src-STAT3 interaction and activation (Fig. 4).

How exactly the c-Src-STAT3 axis promotes breast cancer is not clear but may involve an array of cellular processes including proliferation, survival, epithelial mesenchymal transition (EMT) and tumor formation [47], [67]. Muc1 and VEGF are two proteins regulated by STAT3 which promote invasion and angiogenesis [68]. We have found that transfection of c-Src results in the activation of STAT3 and subsequent induction of Cxcr4, Muc1 and VEGF protein expression and increased breast cancer cell migration, events, which are negated by RKIP over expression (Fig. 4). These results demonstrate that RKIP over expression can inhibit the expression of proteins that are associated with cancer cell invasion and angiogenesis that are regulated by c-Src as well as Src-mediated breast cancer cell migration.

The article "Raf Kinase Inhibitor Protein (RKIP) Blocks Signal Transducer and Activator of Transcription 3 (STAT3) Activation in Breast and Prostate Cancer" was retracted in 2021. Reasons: manipulated images; duplicated images; original data or images not available; unreliable data.

The critical roles played by c-Src and STAT3 in cancer progression make them attractive targets for cancer therapies. RKIP can simultaneously induce apoptosis and migration and inhibit cell-survival pathways, including c-Src-STAT3, in human cancer cells (Figs. 1,3 and 4). We present evidence here that RKIP can suppress signaling pathways leading to cell proliferation which suggests that RKIP may be able to inhibit angiogenesis and metastasis of invasive tumors. There is a clear association between poor prognosis for patients with tumors and low expression levels of RKIP. Treatment with chemotherapeutic agents that induce RKIP expression [29] and/or increase RKIP levels may improve therapeutic outcome for patients with some cancers.

STAT3 is activated in numerous human tumors including breast cancer [7] and has been a target for anticancer therapy [3], [5], [69]. Osteopontin (OPN), a chemokine-like extracellular matrix-associated protein, regulates STAT3 activation that leads to tumor progression and inhibits apoptosis in breast cancer cells [70]. In contrast, inhibition of the STAT3 signaling pathway using JAK-specific inhibitors significantly suppresses the growth of breast cancer cells [71]. Several small molecules have been identified that directly block STAT3 signaling, and their potency and specificity are being investigated [72], [73]. Small compounds that block STAT3 signaling through inhibition of Src activity and induce apoptosis of human breast cancer cells are also under investigation [74], [75]. STAT3 has been shown to be activated in over 50% of breast tumors, primarily through the IL-6/gp130/JAK pathway [63], [64], [76]. Our results indicate that RKIP inhibits c-Src and IL-6-mediated STAT3 activation and tumor formation in breast cancer cells (Figs. 1,4 and 5). Significantly, stable over expression of RKIP attenuates, while ablation of RKIP enhances, IL-6 mediated STAT3 activation (Fig. 5). Given that STAT3 activation requires both tyrosine phosphorylation by IL-6 and JAK and serine phosphorylation by MAPK (Raf-dependent), RKIP is a logical inhibitor of STAT3 activity. Therefore, our data indicate that RKIP behaves as an inhibitor of multiple pathways leading to STAT3 activation. It has been suggested that inhibition of STAT3 activation by interfering with IL-6/gp130/JAK signaling pathway may be an important therapeutic modality in breast cancer [76]. We have shown that RKIP can significantly inhibit activated STAT3-mediated MDA breast cancer cell tumor xenograft growth (Fig. 5). Given the realization of the critical roles played by c-Src and STAT3 in cancer progression, it is imperative to identify agents to antagonize their function. Clearly, RKIP represents a protein that can simultaneously induce apoptosis, inhibit cell survival pathways and tumor growth, including STAT3, in human breast cancer cells.

The article "Raf Kinase Inhibitor Protein (RKIP) Blocks Signal Transducer and Activator of Transcription 3 (STAT3) Activation in Breast and Prostate Cancer" was retracted in 2021. Reasons: manipulated images; duplicated images; original data or images not available; unreliable data.

## Conclusions

RKIP plays a critical role in opposing the effects of pro-oncogenic STAT3 activation. It is not surprising that expression of RKIP may be down regulated during tumor progression. There is a clear association between poor prognosis of a tumor and low expression levels of RKIP [30]–[36]. Suppression of prostate and breast cell survival pathways by RKIP, as demonstrated in this study, indicates the potential ability of enhanced levels of RKIP to inhibit angiogenesis and the metastatic capabilities of invasive tumors. Also, loss of sensitivity to the apoptotic effects of MTIs can be restored by increased RKIP expression. Thus, it may be important to consider the use of chemotherapeutic agents, which induce RKIP expression [29] and/or identify novel compounds to increase RKIP levels in order to improve therapeutic outcome. Identifying molecular mechanisms that antagonize STAT3 activation (in this case, via RKIP) will be very informative for breast and prostate cancer therapy. Further evaluation of RKIP/STAT3 axis in breast/prostate cancer progression is warranted and may provide insight into a novel and important therapeutic approach for the treatment of these diseases.
